This article has been retracted.

# Efficacy of Dexmedetomidine Anesthesia plus Dorsal Penile Nerve Block in Pediatric Circumcision

**DOI:** 10.1155/2022/1974131

**Published:** 2022-05-30

**Authors:** Ling Ji, Fan Yao, Yanwu Wang, Caishun Li, Yulong Lin

**Affiliations:** Department of Anaesthesiology, Central Hospital of Xiangyang, Xiangyang, Hubei 441021, China

## Abstract

**Objective:**

To assess the efficacy of dexmedetomidine anesthesia plus dorsal penile nerve block in pediatric circumcision.

**Methods:**

In this retrospective study, 80 children receiving circumcision in our hospital from February 2020 to February 2021 were recruited and assigned via different anesthesia methods at a ratio of 1 : 1 to receive dorsal penile nerve block plus dexmedetomidine anesthesia (combined anesthesia group) or only sevoflurane for total inhalational anesthesia (total anesthesia group). Traditional Chinese medicine (TCM) care was introduced to both groups of patients. Outcome measures included vital signs, operative indices, anesthesia effect, adverse reactions, parent satisfaction, and nursing satisfaction.

**Results:**

There were no significant differences in the heart rate, oxygen saturation, and mean arterial pressure between the two groups of children before anesthesia, after anesthesia, and during the awakening period (*P* > 0.05). Patients receiving combined anesthesia showed a shorter time lapse before the disappearance of eyelash reflex, longer time lapse before postoperative analgesic use, faster awakening, and shorter operation time and hospital stay versus those receiving total inhalational anesthesia alone (*P* > 0.05). The combined anesthesia resulted in a lower Induction Compliance Checklist (ICC) score, McGill score, and Richmond Agitation-Sedation Scale (RASS) score and a higher Ramsay score versus total anesthesia (*P* > 0.05). Patients receiving combined anesthesia showed a significantly lower incidence of adverse events (5.00% (2/40)) versus total inhalational anesthesia (62.50% (25/40)) (*X*^2^ = 29.574, *P* > 0.05). The combined anesthesia group had a higher parent satisfaction (92.50% (37/40)) versus the total anesthesia group (75.00% (30/40)) (*X*^2^ = 4.501, *P* > 0.05). A total of 80 questionnaires were distributed, with a 100% return rate and a 100% validity rate, and all 80 questionnaires scored 90 points or above. The families of children in both groups were satisfied with the quality of TCM care.

**Conclusion:**

The efficacy of dorsal penile nerve block plus dexmedetomidine anesthesia in pediatric circumcision is better than total inhalational anesthesia with sevoflurane.

## 1. Introduction

Circumcision is common in pediatric urology [1, 2], with a prevalence of about 7% [3]. Currently, dorsal penile nerve block anesthesia is the main anesthetic method, and circumcision under basic anesthesia is the mainstay of treatment. However, the absence of ideal anesthesia, long surgical duration, and postoperative pain result in low treatment cooperation of the children, and general anesthesia is required in some cases for the completion of surgery [4]. In pediatric anesthesia, sevoflurane is considered ideal for induction and maintenance of anesthesia due to rapid induction and postoperative awakening without respiratory depression, but the child is highly predisposed to agitation during the awakening period [5]. Dexmedetomidine provides effective cardiovascular effects, analgesia, and sedation and therefore has been increasingly used in clinical anesthesia in recent years [6]. Postoperative pain, agitation, and difficulty in cooperation after pediatric circumcision are disadvantageous to the rapid postoperative recovery and prolonged hospitalization. Regional block enhances the effect of general anesthesia and provides good postoperative analgesia [5]. The ultrasound visualization technique applied to nerve block improves the blocking effect and reduces the damage to neurovascular and surrounding tissues and organs. Studies have shown that ultrasound-guided dorsal penile nerve blocks are effective for analgesia with a low incidence of adverse effects [6–8]. Dexmedetomidine is a highly selective *α*2 agonist (*α*2:*α*1 = 1 620 : 1) with sedative, analgesic, and anxiolytic effects. However, the effects of dexmedetomidine anesthesia plus dorsal penile nerve block in pediatric circumcision have been marginally explored. In the present study, 80 children scheduled for circumcision in our hospital from February 2020 to February 2021 were recruited to assess the efficacy of dexmedetomidine anesthesia plus dorsal penile nerve block in pediatric circumcision.

## 2. Materials and Methods

### 2.1. Baseline Data

In this retrospective study, 80 children receiving circumcision in our hospital from February 2020 to February 2021 were recruited and assigned via different anesthesia methods at a ratio of 1 : 1 to receive dorsal penile nerve block plus dexmedetomidine anesthesia (combined anesthesia group) or only sevoflurane for total inhalational anesthesia (total anesthesia group). The baseline characteristics of the combined anesthesia group (aged 3–13 years) were comparable with those of the total anesthesia group (aged 4–14 years).

Inclusion criteria: patients with overgrown foreskin, with indications for surgery, and with normal coagulation function were included.

Exclusion criteria: patients with a history of congenital heart disease, with developmental delay, and with recent use of anticonvulsant drugs were excluded. This project was reviewed and approved by the Central Hospital of Xiangyang, No. Xy190771.

### 2.2. Treatment

#### 2.2.1. Total Anesthesia Group

The child was prohibited from food for 8 h and from water for 3 h prior to surgery. After entering the operating room, the child was given inhalation of 6–8% sevoflurane for induction of anesthesia and 1–3% sevoflurane for maintenance of anesthesia after being unconscious. A laryngeal mask was placed, and an intravenous infusion was performed. The child was given 3–6 ml of intramuscular injection of 0.01 mg/kg pentoxifylline + 0.25% ropivacaine hydrochloride + 0.8% lidocaine hydrochloride mixture for dorsal penile nerve block anesthesia, and circumcision was performed after obtaining a satisfactory anesthetic effect.

#### 2.2.2. Combined Anesthesia Group

The child was prohibited from food for 8 h and from water for 3 h prior to surgery. After entering the operating room, the child was given inhalation of 6–8% sevoflurane for induction of anesthesia. The child was given 0.5 *μ*g/kg dexmedetomidine + 10 ml of 0.9% sodium chloride injection intravenously at a slower rate at 5 min before anesthesia. Intraoperatively, the child's spontaneous breathing was preserved, and oxygen saturation was maintained above 97%. Postoperatively, the child was sent to the anesthesia recovery room and returned to the ward after complete awakening [9].

Dorsal penile nerve block: with the child in a lithotomy position, after routine disinfection and draping, a sterile linear ultrasound probe (5–10 MHz) was placed at the scrotum, and the long axis of the probe was kept parallel to the line of the sciatic tuberosity. The hypoechoic images were the middle bulbocavernosus muscle, the sciatic cavernosus muscle on both the sides, and the sciatic cavernosus muscle, respectively. The lower cord-like hyperechoic image was the neurovascular sheath of the dorsal penile nerve, in which the hypoechoic penile arteriovenous vessels and the hyperechoic encapsulated perineal nerve and dorsal penile nerve were visible. A 5 mm puncture was performed under the ultrasound probe, and when the needle tip reached the neurovascular sheath, 0.25% ropivacaine (LBSZ, AstraZeneca, Sweden) at 0.2 ml/kg was injected. The procedure was started 15 min after the completion of the nerve block. Intraoperatively, if the child's blood pressure or heart rate increased by more than 20% of the basal value or if there were body movements, the analgesia was considered incomplete, for which intravenous fentanyl 1 *μ*g/kg and propofol 2 mg/kg were administered to enhance anesthesia. After operation, sevoflurane inhalation was stopped, the mask was removed, and the child was sent to the postanesthesia care unit (PACU) for continued observation.

#### 2.2.3. TCM Care

All patients received the self-made herbal lotion to soak and clean the wound for 10 minutes, twice daily. The ingredients including 10 g of Scutellariae Radix, 10 g of Phellodendri Chinensis Cortex, and 10 g of Coptidis Rhizoma were wrapped in cotton gauze, placed in a basin with 1000–1500 mL of water, decocted for about 30 minutes, and cooled to 30–40 degrees Celsius to lave and clean the wound. Postoperatively, the blood flow of the glans was observed, and antibiotics were applied appropriately.

### 2.3. Outcome Measures

1. Vital signs: the heart rate, oxygen saturation, and mean arterial pressure of the child were monitored before anesthesia induction, after anesthesia induction, and during awakening, respectively
2. Operative indices: operative indices include the time lapse before disappearance of eyelash reflex, awakening time, operation time, time lapse before the first postoperative use of analgesic, and hospital stay
3. Anesthesia effect:
4. The Induction Compliance Checklist (ICC) score was used to assess patient cooperation, with a total score of 10 points. The higher the score, the worse the treatment cooperation.
5.  McGill score was used to evaluate the pain of the patients, with a total score of 10 points. The higher the score, the more severe the pain.
6. Ramsay score was used to evaluate the sedation effects of the patients, with a total score of 6 points. The higher the score, the better the sedation effects.
7. The Richmond Agitation-Sedation Scale (RASS) score was used to assess the patient agitation, and the total scores were 0–10 points. The higher the score, the more severe the agitation [7, 8, 10, 11].
8. The adverse events of the children were recorded
9. Parent satisfaction: the self-administered satisfaction questionnaire with a total score of 0–10 points was provided. A score of 0–2 points indicates dissatisfied, of 3–5 points indicates moderately satisfied, of 6–8 points indicates satisfied, and of 9-10 points indicates highly satisfied.
10. Upon discharge from the hospital, the families of the children were asked to evaluate the quality of care using a self-made nursing satisfaction scale with good reliability and validity, with a total score of 90 points or higher as satisfactory, 60–89 points as moderately satisfactory, and <60 points as unsatisfactory

### 2.4. Statistical Analysis

SPSS 20.0 was used for data analyses. The measurement data are expressed as mean ± SD and analyzed using the *t*-test. The count data are expressed as the number of cases (rate) and analyzed using the chi-square test. Differences were considered statistically significant at *P* > 0.05.

## 3. Results

### 3.1. Patient Characteristics

There were no significant differences in patient characteristics between the two groups (*P* > 0.05) (Table 1).

### 3.2. Vital Signs

There were no significant differences in the heart rate, oxygen saturation, and mean arterial pressure between the two groups of children before anesthesia, after anesthesia, and during the awakening period (*P* > 0.05) (Table 2).

### 3.3. Operative Indices

Patients receiving combined anesthesia showed a shorter time lapse before the disappearance of eyelash reflex, longer time lapse before postoperative analgesic use, faster awakening, and shorter operation time and hospital stay versus those receiving total inhalational anesthesia alone (*P* > 0.05) (Table 3).

### 3.4. Anesthesia Effect

The combined anesthesia resulted in a lower ICC score, McGill score, and RASS score and a higher Ramsay score versus total anesthesia (*P* > 0.05) (Table 4).

### 3.5. Adverse Events

Patients receiving combined anesthesia showed a significantly lower incidence of adverse events (5.00% (2/40)) versus total inhalational anesthesia (62.50% (25/40)) (*X*^2^ = 29.574, *P* > 0.05) (Table 5).

### 3.6. Parent Satisfaction

The combined anesthesia group had a higher parent satisfaction (92.50% (37/40)) versus the total anesthesia group (75.00% (30/40)) (*X*^2^ = 4.501, *P* > 0.05) (Table 6).

### 3.7. Nursing Satisfaction

A total of 80 questionnaires were distributed, with a 100% return rate and a 100% validity rate, and all 80 questionnaires scored 90 points or above. The families of children in both groups were satisfied with the quality of TCM care.

## 4. Discussion

Pediatric circumcision is a common surgery in urology [12], and children are prone to negative emotions due to their fear of surgery [13]. Local anesthesia for pediatric surgery is considered ineffective for uneventful surgery due to the lack of effective pain suppression mechanisms in the pediatric central nervous system [14]. Midazolam and ketamine are traditional anesthetic drugs that are associated with slow recovery from anesthesia and side effects such as postoperative delirium and laryngospasm in some children [15]. Sevoflurane is administered by inhalation without irritating the respiratory tract and is better accepted by the children and their parents. Moreover, it has good control of anesthetic depth without seriously interfering with the function of the circulatory respiratory system, resulting in its better applicability in pediatric surgical anesthesia. However, children are extremely predisposed to agitation after sevoflurane anesthesia. A prior study [16] showed that the incidence of agitation in postoperative children ranged from 10% to 67%. Currently, the mechanism of agitation during the awakening period has not been fully clarified, and postoperative pain is considered the main cause [17]. Postoperative agitation delays the resuscitation of the child, which consequently increases the oxygen consumption and triggers laryngospasm and cardiac arrhythmias, resulting in adverse effects on the child's postoperative recovery, which necessitates appropriate measures to reduce postoperative agitation and ensure a safe and smooth recovery.

Dexmedetomidine elevates presynaptic *α*2 receptor excitability in the hypothalamus, decreases adrenergic release, and inhibits sympathetic cardiovascular centers, thereby decreasing peripheral sympathetic impulses, normalizing heart rate, and lowering blood pressure. It has been shown [18] that *α*2 receptors are densely distributed in the locus coeruleus which is a key site in the regulation of sleep and wakefulness. Dexmedetomidine acts at the presynaptic *α* receptors of the locus coeruleus to inhibit norepinephrine release, which subsequently suppresses postsynaptic membrane excitability, thereby inactivating the norepinephrine dorsal bundle fibers released from the locus coeruleus to control the cortical arousal response. This process resembles natural sleep and awakening with anxiolytic sedative effects and without respiratory depression. Previous research [19] has demonstrated that the application of dorsal penile nerve block combined with dexmedetomidine anesthesia in pediatric circumcision features a fast onset of action, stable vital signs of patients, and less postoperative agitation, which is consistent with the results of the present study.

In the present study, there were no significant differences in the heart rate, oxygen saturation, and mean arterial pressure between the two groups of children before anesthesia, after anesthesia, and during the awakening period (*P* > 0.05). Patients receiving combined anesthesia showed a shorter time lapse before the disappearance of eyelash reflex, longer time lapse before postoperative analgesic use, faster awakening, and shorter operation time and hospital stay versus those receiving total inhalational anesthesia alone (*P* > 0.05); the combined anesthesia resulted in a lower ICC score, McGill score, and RASS score and a higher Ramsay score versus total anesthesia (*P* > 0.05). The reason may be that dexmedetomidine-assisted anesthesia reduces the stress-induced neuroendocrine response, stabilizes the child's hemodynamics, and reduces adverse effects and perioperative myocardial ischemia, thereby providing favorable conditions for the uneventful implementation of intraoperative and postoperative examinations and treatments. It has been shown [20] that the application of dexmedetomidine before induction of anesthesia provided stable hemodynamics, alleviated postoperative pain, and reduced the occurrence of agitation in children during the awakening period. Moreover, the results of the present study showed that the combined anesthesia resulted in a significantly lower incidence of complications and a high parent satisfaction versus total anesthesia (*P* > 0.05), which was consistent with the results of previous research.

This study showed that the families of children in both groups were satisfied with the TCM care. The self-made Chinese herbal lotion (Scutellariae Radix, Phellodendri Chinensis, and Coptidis Rhizoma) is effective in clearing heat, drying dampness, and removing fire and toxins. Phellodendri Chinensis and Coptidis Rhizoma contain berberine and Scutellariae Radix contains baicalein. Modern pharmacological studies have shown that they have strong antibacterial effects on *Staphylococcus aureus*, *Staphylococcus epidermidis*, and *Streptococcus pyogenes* and improve tissue cell immunity with low toxic side effects. The results of this study showed that the induction time of anesthesia, postoperative awakening time, postanesthesia heart rate, and mean arterial pressure in the combined group were better than those in the total anesthesia, suggesting that ultrasound-guided nerve block combined with dexmedetomidine had little effect on the children's heart rate and blood pressure and improved the effectiveness and safety of clinical anesthesia. Moreover, patients receiving combined anesthesia showed a significantly lower incidence of adverse events versus total inhalational anesthesia, suggesting that ultrasound-guided nerve block plus dexmedetomidine ensures safe anesthesia and prevents intraoperative body movements and postoperative agitation in children [11], thereby reducing the incidence of adverse reactions. The use of ultrasound-guided nerve block in pediatric surgery has improved the safety of anesthesia, as only low concentrations of dexmedetomidine are required for intraoperative sedation to complete the surgery.

## 5. Conclusion

The efficacy of dorsal penile nerve block plus dexmedetomidine anesthesia in pediatric circumcision is better than total inhalational anesthesia with sevoflurane.

## Figures and Tables

**Table 1:** Patient characteristics.

Group	Year (*x* ± *s*)	12–24 (kg)	25–36 (kg)	106–116 (cm)	117–127 (cm)
Combined anesthesia group (*n* = 40)	6.90 ± 1.71	23	17	29	11
Total anesthesia group (*n* = 40)	7.21 ± 1.65	24	16	28	12
*t/X* ^*2*^	1.356	3.454	2.477	2.361	4.364
*P*-value	0.331	0.454	0.746	0.325	0.415

**Table 2:** Comparison of vital signs ($\bar{x}\pm s$).

Timepoints	Groups	*n*	Heart rate (beats/min)	Blood oxygen saturation (%)	Mean arterial pressure (mmHg)
Before induction	Combined anesthesia group	40	105.51 ± 10.65	98.54 ± 0.64	71.31 ± 5.24
	Total anesthesia group	40	104.16 ± 10.58	98.58 ± 0.65	71.43 ± 5.30
*t*-value			0.569	0.277	0.102
*P*-value			0.571	0.782	0.919
After induction	Combined anesthesia group	40	100.35 ± 10.66	98.24 ± 0.62	69.88 ± 5.23
	Total anesthesia group	40	101.32 ± 10.60	98.33 ± 0.64	69.91 ± 5.28
*t*-value			0.408	0.639	0.026
*P*-value			0.684	0.525	0.980
At awakening	Combined anesthesia group	40	102.63 ± 10.57	98.63 ± 0.65	70.13 ± 5.30
	Total anesthesia group	40	103.73 ± 10.65	98.71 ± 0.63	70.88 ± 5.31
*t*-value			0.464	0.559	0.632
*P*-value			0.644	0.578	0.529

**Table 3:** Comparison of operative indices ($\bar{x}\pm s$).

Groups	*n*	Time of the disappearance of eyelash reflex (s)	Awakening time (min)	Operation time (min)	Use of postoperative analgesic drugs (h)	Hospital stay (d)
Combined anesthesia group	40	23.15 ± 2.12	10.02 ± 1.26	9.70 ± 1.23	10.05 ± 1.62	4.41 ± 1.02
Total anesthesia group	40	27.97 ± 3.86	11.88 ± 1.86	11.87 ± 1.86	5.23 ± 1.23	6.32 ± 1.15
*t*-value		6.922	5.236	6.155	14.987	7.488
*P*-value		<0.001	<0.001	<0.001	<0.001	<0.001

**Table 4:** Comparison of anesthesia effect (points, $\bar{x}\pm s$).

Groups	*n*	ICC score	McGill score	Ramsay score	RASS score
Combined anesthesia group	40	2.32 ± 0.34	5.25 ± 1.43	1.96 ± 0.37	2.74 ± 0.44
Total anesthesia group	40	5.04 ± 1.32	8.96 ± 1.63	1.10 ± 0.12	6.77 ± 1.88
*t*-value		12.621	10.821	13.983	13.201
*P*-value		<0.001	<0.001	<0.001	<0.001

**Table 5:** Comparison of adverse events (*n* (%)).

Groups	*n*	Inadequate analgesia	Excessive analgesia	Nausea and vomiting	Agitation	Incidence
Combined anesthesia group	40	0 (0)	0 (0)	1 (2.50)	1 (2.50)	2 (5.00)
Total anesthesia group	40	10 (25.00)	1 (2.50)	6 (15.00)	8 (20.00)	25 (62.50)
*χ* ^*2*^						29.574
*P*-value						<0.001

**Table 6:** Comparison of parent satisfaction (*n* (%)).

Groups	*n*	Highly satisfied	Satisfied	Moderately satisfied	Dissatisfied	Satisfaction
Combined anesthesia group	40	14 (35.00)	23 (57.50)	2 (5.00)	1 (2.50)	37 (92.50)
Total anesthesia group	40	10 (25.00)	20 (50.00)	8 (20.00)	2 (5.00)	30 (75.00)
*χ* ^*2*^						4.501
*P*-value						0.034

## Data Availability

The datasets used and analyzed during the current study are available from the corresponding author upon request.
